# MicroRNA-34c Inhibits Osteogenic Differentiation and Valvular Interstitial Cell Calcification via STC1-Mediated JNK Pathway in Calcific Aortic Valve Disease

This article has been retracted.

**DOI:** 10.3389/fphys.2020.00829

**Published:** 2020-08-31

**Authors:** Lieming Yang, Xinyuan Zhu, Yingying Ni, Dawei Wu, Yikui Tian, Zhi Chen, Mingbiao Li, Hao Zhang, Degang Liang

**Affiliations:** Department of Cardiovascular Surgery, Tianjin Medical University General Hospital, Tianjin, China

**Keywords:** MicroRNA-34c, stanniocalcin 1, c-Jun N-terminal kinase (JNK), osteogenic differentiation, calcified aortic valve

## Abstract

Calcific aortic valve disease (CAVD), a common heart valve disease, is increasingly prevalent worldwide and causes high morbidity and mortality. Here, we aimed to investigate a possible role for miR-34c in the development of osteogenic differentiation during CAVD and to find out the underlying mechanisms. Valvular interstitial cells (VICs) were isolated from the clinical aortic valve tissue samples of CAVD patients and patients with acute aortic dissection and collected. Then, RT-qPCR was performed to determine miR-34c expression and western blot analysis was applied to confirm the relevant protein expression in these VICs. Dual luciferase reporter gene assay was applied to confirm the relation between miR-34c and STC1. Alkaline phosphatase (ALP) staining and alizarin red staining was performed to further confirm the degree of calcification in these samples. MiR-34c was lowly expressed and STC1 was highly expressed in the CAVD tissues. Furthermore, STC1 was the target of miR-34c and was negatively regulated by miR-34c. Overexpression of miR-34c in VICs was concomitant with suppression of both STC1 expression and phosphorylation level of c-Jun N-terminal kinase (JNK). In addition, significant decrease of bone morphogenetic protein-2 (BMP2) and osteocalcin, as well as the decrease of calcification degree were also observed in VICs with miR-34c overexpressed. Taken together, miR-34c could inhibit osteogenic differentiation and calcification of VICs by suppressing the STC1/JNK signaling pathway in CAVD, making miR-34c a novel therapeutic target for the treatment of CAVD.

## Introduction

Calcific aortic valve disease (CAVD) is one of the most prevalent heart diseases associated with high morbidity and mortality, whose incidence increases when the population ages (Yutzey et al., 2014; Hulin et al., 2018). CAVD consists of two syndromes, namely, changes in lobular cells firstly and then a terminal calcification which leads to the obstruction of the left ventricular outflow tract (Rajamannan et al., 2011). Several factors, including age and smoking, may increase the risk of this disease (Towler, 2013). Valvular interstitial cells (VICs) are responsible for secretion and remodeling the valvular tissue matrix, thus modulating the balance between homeostasis and disease (Mabry et al., 2015).

MicroRNAs (miRNAs) are short, single-stranded, non-coding RNA approximately 20–25 nucleotides in length. miRNAs play important roles in regulating various biological processes, including proliferation, apoptosis, and differentiation (Bouhallier et al., 2010). For instance, miRNAs can change the phenotype of VICs when flow is disturbed during aortic stenosis (Oury et al., 2016). In addition, increasing evidence showed that miRNAs could play a role in the treatment of cardiovascular diseases, such as heart failure (Vegter et al., 2016). A previous study found that 92 miRNAs were differentially expressed in CAVD patients compared with healthy controls, and the differential expression of miRNAs was correlated with several different targets and pathways (Wang et al., 2017). For example, one study confirmed that miR-101b targeted ataxin-1 and stanniocalcin-1 (STC1) (De Martino et al., 2009).

STC1, a STC mammalian homolog and considered to be a homodimeric phosphoglyco-protein, was firstly identified in fish bone to mediate the production of calcium/phosphate calcium (Yoshiko and Aubin, 2004), calcium phosphate homeostasis and to preserve against hypercalcemia in fish bone (Zhang et al., 2000). In liver cancer, high expression of STC1 resulted in reduced energy metabolism, thus culminating in an activation of the AMPK pathway but a blockage of p70/p-rpS6 pathway to reduce tumor growth (Leung and Wong, 2018). In cervical cancer, STC1 regulates cell apoptosis via the NF-κB phospho-P65 Ser536 pathway (Pan et al., 2017). STC1 can prevent the accumulation of excessive cytosolic Ca2^+^ to protect cardiomyocytes from damage, and it also regulates endothelial functions in failing heart (Koizumi et al., 2007) and cardiovascular inflammation (Chen et al., 2008). *In vitro* analysis of aortic vascular smooth muscle cells showed that inorganic phosphate induction significantly enhanced mRNA expression of STC2 and osteocalcin (Takei et al., 2012), implying the possible positive correlation between STC2 and osteocalcin. Furthermore, another study found that secretion of STC1 might lead to potential metastasis of hepatocellular carcinoma by regulating the JNK pathway (Chan et al., 2017). Another study indicated that aberrant STC1 could enhance triple-negative breast cancer cell invasive ability via the JNK pathway (Han et al., 2016). JNK is a kinase with multiple functions and plays a role in various physiological and pathological processes. Therefore, we hypothesized that miR-34c may mediate osteogenic pathway by STC1 gene-mediated JNK pathway to affect aortic valve calcification.

## Materials and Methods

### Ethics Statement

The studies involving human participants were reviewed and approved by Institutional Review Board of Tianjin Medical University General Hospital. The patients/participants provided their written informed consent to participate in this study.

### Bioinformatic Analysis

The microarray datasets GSE77287 of CAVD were retrieved from the Gene Expression Omnibus database^1^. R language was used for screening differentially expressed gene analysis with |log (fold change)| > 1 and *p value* < 0.05 as threshold values.

### Clinical Sample Collection

Tissue samples were collected form 32 patients (mean age: 69.47 ± 9.02 years old) pathologically diagnosed as CAVD and admitted in Tianjin Medical University General Hospital from June 2017 to December 2018. These patients consisted of 19 males and 13 females. None of them had congenital malformation of heart valves or rheumatic valvular disease. In addition, control aortic valve (normal AV) from another 25 age-matched patients with acute aortic dissection were collected as a common, which consisted of 14 males and 11 females. Both the CAVD and the AV tissue samples were collected and kept frozen at −80°C until further use.

### Extraction of Valve Interstitial Cells (VICs)

Valve Interstitial Cells were isolated from patients with acute aortic dissection under sterile conditions. After extensive washes with 0.1 mL of phosphate-buffered saline, the valve leaflets were lightly scraped with a blade at the surface for two to three times. After removal of endothelial cells, the leaflets were detached with Dulbecco’s modified Eagle’s medium (DMEM) containing high concentration of glucose (Gibco, Carlsbad, CA, United States) and 2 mg/mL type I collagenase (Sigma-Aldrich Corporation, Missouri, United States) for 8 h at 37°C. After vortexing and repeated aspirating to break up the tissue mass, the suspension was filtered through a 100 μm mesh screen and subsequently centrifuged at 1500 rpm for 3 min. Afterward, primary human VICs were acquired by resuspending the centrifuged pellet in 5 mL high glucose DMEM containing 10% fetal bovine serum (FBS). Cells at passage 3 were used for all experiments.

### Culture of Osteoblasts

Valve Interstitial Cells were seeded in 24-well plates at a density of 2 × 10^5^ cells/well. The cells were maintained in 0–500 ng/mL recombinant human NELL-1 or 100 ng/mL recombinant human bone morphogenetic protein-2 (BMP2) in the presence of osteogenic media (OM) containing DMEM, 10% FBS (Gemini, Woodland, CA, United States), 50 lg/mL ascorbic acid, 10 mM b-glycerol phosphate, 10^–8^ dexamethasone. The culture medium was supplemented every 3 days for 2 weeks.

### Cell Treatment

Valve Interstitial Cells were subjected to the following treatments: negative control (NC) mimic plasmid (5′-AGCG UGCCUGAGCAUAGGUGAU-3′), miR-34c mimic (5′-AGUGA CGGUGAGCUUAGCUGAU-3′), miR-34c inhibitor (5′-AUCAC CUAUGCUCAGGCACGCU-3′); NC inhibitor plasmid (5′-AU GAGCAAUCCACUGCCUGGCA-3′), overexpressed (oe)-NC plasmid, oe-stanniocalcin 1 (STC1), 10 mmol/L dimethyl sulfoxide (DMSO), 10 mmol/L c-Jun N-terminal kinase (JNK) inhibitor SP600125 (HY-12041, MedChemExpress, Shanghai, China) alone or in combination. pCMV6-AC-GFP (overexpression plasmid) and pGPU6/Neo (silencing plasmid) were purchased from Fenghui Biotechnology Co., Ltd. (FH1215, Changsha, Hunan, China) and Shanghai GenePharma Co., Ltd. (Shanghai, China), respectively. After 24 h of cell culture, transient transfection was conducted using Lipofectamine 2000 (11668-019, Invitrogen, New York, CA, United States) according to the manufacturer’s instructions, and 48 h later, the following experiments were carried out.

### Reverse Transcription Quantitative Polymerase Chain Reaction (RT-qPCR)

Total RNA was extracted from cells (24 h after transfection) and tissues using TRIzol (Invitrogen, Carlsbad, CA, United States) and reverse transcribed into complementary DNA (cDNA) according to the specifications of TaqMan MicroRNA Assays Reverse Transcription Kit (4427975, Applied Biosystems, Foster City, CA, United States). Primers for miR-34c (Table 1) were synthesized by Takara Bio Inc (Kyoto, Japan). Then RT-qPCR was performed using an ABI7500 quantitative PCR instrument (7500, Applied Biosystems, Foster City, CA, United States). U6 was used as an internal reference for the quantity of miR-34c. The relative transcription level of the target gene was calculated by Relative quantification (2^–ΔΔ*CT*^ Method).

**TABLE 1:** Primer sequences for RT-qPCR.

	**Primer sequences (5′-3′)**
miR-34c	F: 5′-GCTGCTGTAGGCAGTGTAGTTAG-3′ R: 5′-CTCAACTGGTGTCGTGGAGTC-3′
U6	F: 5′-CTCGCTTCGGCAGCACA-3′ R: 5′-AACGCTTCACGAATTTGCGT-3′

*RT-qPCR, reverse transcription quantitative polymerase chain reaction; F, forward; R, reverse; miR-34c, microRNA-34c.*

### Western Bolt Analysis

Total protein was isolated from tissues or cells (48 h after transfection) using radioimmunoprecipitation assay buffer. The protein was separated by the sodium dodecyl sulfate-polyacrylamide gel electrophoresis. Afterward, proteins were transferred to a polyvinylidene fluoride (PVDF) membrane, and then blocked with 5% skim milk powder at room temperature for 1 h. Subsequently, the PVDF membrane was incubated with the corresponding diluted antibody overnight at 4°C. The following primary antibodies were used: rabbit antibodies to STC1 (1:1000, ab83065, Abcam, Cambridge, United Kingdom); p-JNK (1:1000, ab124956, Abcam); JNK (1:2000, ab208035, Abcam); bone morphogenetic protein-2 (BMP2; 1:1000, ab14933, Abcam). Osteocalcin (1:500, ab93876, Abcam). Glyceraldehyde-3-phosphate dehydrogenase (GAPDH; ab9485, 1:2500) was used as a normalization medium. The blot was incubated with horseradish peroxidase-conjugated goat anti-rabbit immunoglobulin G (IgG) secondary antibody (ab97051, 1:2000, Abcam) for 1 h. Protein bands were visualized using the enhanced chemiluminescence detection kit (No. BB-3501, Amersham Pharmacia Biotech, Chicago, IL, United States) and Bio-Rad Image analysis system (Bio-Rad Laboratories, Inc., Hercules, CA, United States). Software Quantity One v4.6.2 was used for the further quantifying analysis.

### Dual Luciferase Reporter Gene Assay

The STC1-Wild type (STC1-Wt) cDNA fragments, containing 3′-untranslated region (UTR) (the binding site of miR-34c) were inserted into the pmirGLO vector. The, STC1-mutant (STC1-Mut) cDNA fragments, with the 3′-UTR mutated was inserted into pmirGLO vector. The insertion sequence was verified by sequencing (The above operation was completed by Shanghai RiboBio Co., Ltd., Shanghai, China). Then, pmirGLO-STC1-Wt or pmirGLO-STC1-Mut recombinant vectors were co-transfected into HEK293T cells with miR-34c mimic or miR-NC mimic using the Liposome transfection method. After transfection and further culture for 48 h, cells were lysed and then the supernatant was collected as samples for detection. The activity of renilla luciferase was determined using multiscan spectrum SpectraMax M5 (Molecular Devices, Shanghai, China).

### Alizarin Red Staining

Valve Interstitial Cells were induced by OM for 14 days and then stained by alizarin red. VICs were fixed with 95% ethyl alcohol for 15 min. After incubation with alizarin red solution for 5 min, excessive dye was removed by washing with distilled water. VICs were mounted after air-drying. The microscope (Carl Zeiss AG, Jena, Germany) was used to observe calcified nodules in VICs after different treatments.

### Alkaline Phosphatase (ALP) Staining

The VICs were induced by OM for 14 days and then stained using the ALP stain kit (1102-100, Innovative Cellular Therapeutics, Shanghai, China) in the dark at room temperature for 15 min. After that, cells were washed with distilled water for 2–3 times to terminate the reaction. At last, the microscope (Carl Zeiss AG, Jena, Germany) was used to observe staining in VICs after different treatments. ALP activity was measured using an ALP detection kit (Nanjing Jiancheng Bioengineering Institute, Nanjing, Jiangsu, China).

### Statistical Analysis

Statistical analysis was conducted using SPSS 21.0 statistical software (IBM Corp. Armonk, NY, United States). Measurement data were presented as mean ± standard deviation. Differences between two groups were compared by unpaired Student’s *t* test if data were in normal distribution. Comparison among multiple groups was conducted by one-way analysis of variance (ANOVA) and Tukey *post hoc* test. *P* < 0.05 was used to indicate a statistical significance.

## Results

### Down-Regulated Expression of miR-34c Is Found in Calcified Aortic Valves (AVs)

A previous study found that miR-34c expression was down-regulated in calcified vascular smooth muscle cells (Hao et al., 2016). In this study, clinical samples from patients with CAVD and patients with acute aortic dissection were collected to investigate the expression of miR-34c in calcified AV. RT-qPCR was used to determine the expression of miR-34c in the arterial flap of these tissue samples and the result showed a relatively lower expression of miR-34c in CAVD compared to normal AV tissues from acute aortic dissection patients (Figure 1).

**FIGURE 1:** The expression of miR-34c is downregulated in calcified AV. The expression of miR-34c in tissue samples of arterial flap was determined by RT-qPCR. Data are presented as mean ± standard deviation. Differences between negative control (*n* = 32) and CAVD group (*n* = 25) are compared using the unpaired Student’s *t* test.

### MiR-34c Inhibits Osteogenic Differentiation and Calcification of VICs

To further explore the functional role of miR-34c during CAVD in VIC, VICs were extracted from CAVD tissues and transfected with either miR-34c mimic plasmid or miR-34c inhibitor plasmids to achieve the gain-of-function and lost-of-function studies. The expression of miR-34c in the different transfected groups was confirmed by RT-qPCR. The results showed that miR-34c expression was upregulated in VICs transfected with miR-34c mimic (*p* < 0.05), while the expression decreased significantly in VICs transfected with miR-34c inhibitor group compared to VICs transfected with NC mimic plasmid (*p* < 0.05; Figure 2A). The expression of BMP2 and bone cell differentiation marker protein, osteocalcin, was measured using western blot analysis. We found that the expression of BMP2 and osteocalcin was decreased markedly in VICs transfected with miR-34c mimic (*p* < 0.05) but increased significantly in VICs transfected with miR-34c inhibitor (*p* < 0.05; Figure 2B).

**FIGURE 2:** Inhibition of miR-34c expression suppresses osteogenic differentiation and VICs calcification. VICs were transfected with NC mimic plasmid, miR-34c mimic, NC inhibitor plasmid or miR-34c inhibitor. **(A)** miR-34 expression measured by RT-qPCR in VICs after different transfection treatment. **(B)** Protein expression of BMP2 and osteocalcin measured by western blot analysis in VICs after different transfection treatment. **(C)** Alizarin red staining (×200) for calcification in VICs after different transfection treatment. **(D)** ALP staining (×200) and quantitative ALP activity analysis in VICs after different transfection treatment. Data are expressed as mean ± standard deviation from at least three independent experiments. The comparison between two groups was checked by unpaired Student’s *t* test. *p < 0.05 vs. VICs transfected with NC mimic. ^#^*p* < 0.05 vs. VICs transfected with NC inhibitor.

In addition, the alizarin red staining indicated that VICs transfected with miR-34c mimic exhibited a significant reduction in the formation of calcified nodules compared with VICs transfected with controls as less red staining spots were found (*p* < 0.05). In contrast, the staining was darker in VICs transfected with miR-34c inhibitor, which suggested a significant increase in the formation of calcified nodules (*p* < 0.05; Figure 2C). VICs transfected with miR-34c mimic suppressed ALP activity and exhibited lighter ALP staining than VICs transfected with controls (*p* < 0.05). On the other hand, darker ALP staining was observed in VICs transfected with miR-34c inhibitor indicating an increase in ALP activity (*p* < 0.05; Figure 2D). Taken together, osteogenic differentiation and calcification of VICs could be inhibited by miR-34c.

### STC1 Is Downregulated by miR-34c

To understand the mechanism of action of miR-34c in CAVD, the target genes of miR-34c were predicted using the miRNA-mRNA online database, miRmap (Figure 3A). Together with the findings of the upregulated genes in CAVD-associated GSE77287 dataset (Figure 3B), the scope of potential target genes was narrowed down to one gene, that is STC1. Firstly, based on the online prediction, STC1 was found to own binding sites with miR-34c. Furthermore, western blot analysis showed that STC1 expression was higher in samples of CAVD compared to normal AV samples (*p* < 0.05; Figure 3C). Dual luciferase reporter gene assay was used to examine the potential interaction between miR-34c and STC1 in HEK293T cells. The results showed decreased luciferase activity in VICs co-transfected with miR-34c mimic and STC1-Wt in comparison with VICs co-transfected with NC mimic and STC1-Wt (*p* < 0.05). In contrast, there was no significant difference in luciferase activity in VICs transfected with STC1-Mut, which revealed that miR-34c could specifically bind to STC1 (Figure 3D).

**FIGURE 3:** The expression of STC1 is downregulated by miR-34c. **(A)** intersection between target genes predicted by the miRmap database (score > 95) and genes highly expressed in calcified AV in GSE77287. **(B)** Volcano plot of differentially expressed genes in microarray datasets GSE77287 of calcified AV. The downregulated genes were presented in green dots and upregulated genes were presented in red dots. The triangle represented the gene STC1. **(C)** Protein expression of STC1 in clinical AV samples determined by western blot analysis. Data are presented as mean ± standard. The comparison between negative control (*n* = 32) and CAVD (*n* = 25) was checked by unpaired Student’s *t* test. **(D)** Dual luciferase reporter gene assay to verify the correlation between miR-34c and STC1. **(E)** Protein expression of STC1 measured by western blot analysis after the overexpression or silencing of miR-34c in VICs. Data were presented as mean ± standard deviation from at least three independent experiments. Comparison between two groups was checked by unpaired Student’s *t* test. ^∗^*p* < 0.05 vs. negative control clinical samples. ^#^*p* < 0.05 vs. VICs transfected with NC mimic. ^&^*p* < 0.05 vs. VICs transfected with NC inhibitor.

In order to study the ability of miR-34c to regulate STC1 expression, STC1 expression was measured by western blot analysis after overexpressing or silencing miR-34c in VICs. STC1 expression was downregulated in VICs transfected with miR-34c mimic, compared with VICs transfected NC mimic, and the expression of STC1 was upregulated in in VICs transfected with miR-34c inhibitor (*p* < 0.05; Figure 3E). In summary, these results suggested that STC1 is a target gene of miR-34c.

### MiR-34c Inhibits the Osteogenic Differentiation and Calcification of VICs by Targeting STC1

In order to investigate the role of miR-34c in the osteogenic differentiation and calcification of VICs, VICs were transfected with NC mimic + oe-NC, NC mimic + oe-STC1, or miR-34c mimic + oe-STC1, respectively. The expression of STC1 in VICs after transfection was determined by western blot analysis and the results are shown in Figure 4A. STC1 expression was upregulated in NC mimic + oe-STC1 group in comparison with the NC mimic + oe-NC group (*p* < 0.05), which confirmed that the overexpression of STC1 was successfully delivered in this study. Nevertheless, STC1 expression was downregulated when VICs were co-transfected with miR-34c mimic and oe-STC1 compared to NC mimic + oe-STC1 treatment (*p* < 0.05). Next, the effects of STC1 on BMP2 and osteocalcin protein expression were further investigated. As expected, the expression of BMP2 and osteocalcin increased significantly in VICs with NC mimic + oe-STC1 treatment (*p* < 0.05). However, their expression was downregulated markedly in VICs with miR-34c mimic + oe-STC1 treatment compared with VICs transfected with NC mimic + oe-STC1 (*p* < 0.05; Figure 4B).

**FIGURE 4:** The osteogenic differentiation and calcification degree of VICs is inhibited by miR-34c via suppressing the expression of STC1. VICs were transfected with NC mimic + oe-NC plasmid; NC mimic + oe-STC1; and miR-34c mimic + oe-STC1, respectively. **(A)** The protein expression of STC1 in VICs with different treatment measured by western blot analysis. **(B)** The protein expression of BMP2 and osteocalcin determined by western blot analysis. **(C)** Alizarin red staining (×200) of calcification. **(D)** The staining figure of ALP (×200) and ALP quantitative activity analysis. Data were expressed as mean ± standard from at least three independent experiments. The comparison between two groups was checked by unpaired Student’s *t* test. *p < 0.05 vs. VICs transfected with NC mimic + oe-NC. ^#^*p* < 0.05 vs. VICs transfected with NC mimic + oe-STC1.

Similarly, the alizarin red staining was also conducted in these transfected VICs to investigate the function of co-transfecting miR-34c and STC1 on calcified nodule formation. As shown in Figure 4C, the alizarin red staining was relatively darker in the VICs transfected with NC mimic + oe-STC1, suggesting that the calcified nodule formation in VICs was significantly increased (*p* < 0.05). In contrast, the staining was lighter in VICs transfected with miR-34c mimic + oe-STC1 compared with NC mimic + oe-STC1 treatment, which suggested that the formation of calcified nodules in VICs was markedly decreased (*p* < 0.05). In addition, ALP staining showed that VICs with NC mimic + oe-STC1 treatment exhibited a relatively dark staining, and an increased ALP activity (*p* < 0.05). Of note, staining was shallow and ALP activity was decreased significantly in VICs with miR-34c mimic + oe-STC1 treatment compared with NC mimic + oe-STC1 treatment (*p* < 0.05; Figure 4D). The above experiments demonstrated that the overexpression of STC1 could result in osteogenic differentiation and calcification of VICs and yet overexpressed miR-34c could reverse the effects of STC1 overexpression in VICs. In summary, it is suggested that miR-34c could downregulate the expression of STC1, thus mediating the osteogenic differentiation and calcification degree of VICs.

### MiR-34c Inhibits CAVD by Suppressing STC1 and Blocking the JNK Pathway

It has been reported that STC1 could activate the JNK pathway (Chan et al., 2017) and the suppression of the JNK pathway could inhibit osteoblast differentiation (Matsuguchi et al., 2009). We treated VICs with oe-NC, oe-STC1, NC mimic + oe-STC1 or miR-34c mimic + oe-STC1. After 10 min and 48 h later, the extent of JNK phosphorylation was detected by Western blot analysis. There was no difference in the extent of JNK phosphorylation among the four groups at 10 min, as shown in Figure 5A. After 48 h, the extent of JNK phosphorylation was markedly increased in VICs transfected with oe-STC1 in comparison with those transfected with oe-NC (*p* < 0.05). In contrast, it was significantly decreased in VICs transfected with miR-34c mimic + oe-STC1 compared with VICs transfected with NC mimic + oe-STC1 (*p* < 0.05). The results indicate that in VICs, STC1 may facilitate activation of the JNK pathway, while miR-34c may inhibit the activation of JNK pathway by suppressing STC1.

**FIGURE 5:** MiR-34c plays a role in CAVD via mediating JNK pathway by inhibiting STC1. **(A)** The phosphorylation level of JNK pathway in VICs with different treatments evaluated by western blot analysis. **(B)** The protein expression of BMP2 and osteocalcin determined by western blot analysis. **(C)** Alizarin red staining (×200) of calcification. **(D)** The staining figure of ALP (×200) and ALP quantitative activity analysis. Data are expressed as mean ± standard from at least three independent experiments. The comparison between two groups was checked by unpaired Student’s *t* test. *p < 0.05 vs. VICs transfected with oe-NC. ^#^*p* < 0.05 vs. VICs transfected with NC mimic + oe-STC1 or miR-34c inhibitor + DMSO. ^&^*p* < 0.05 vs. VICs treated with oe-STC1 + DMSO.

Valve Interstitial Cells were transfected with oe-NC, oe-STC1, miR-34c inhibitor + DMSO, miR-34c inhibitor + SP600125, oe-STC1 + DMSO or oe-STC1 + SP600125. Then, the protein expression of BMP2 and osteocalcin was determined by western blot analysis. Protein expression of BMP2 and osteocalcin in response to miR-34c inhibitor + SP600125 treatment was decreased when compared with miR-34c inhibitor + DMSO treatment (*p* < 0.05). The treatment of oe-STC1 alone induced BMP2 and osteocalcin expression, while SP600125 treatment could counteract the stimulative effect of oe-STC1 on BMP2 and osteocalcin expression (*p* < 0.05; Figure 5B).

The faint staining of the alizarin red and the decreased calcified nodule formation occurred after treatment with miR-34c inhibitor + SP600125 compared with miR-34c inhibitor + DMSO treatment (*p* < 0.05). Similar results also occurred in VICs transfected with oe-STC1 + SP600125 treatment compared with oe-STC1 + DMSO treatment (*p* < 0.05). By contrast, overexpression of STC1 contributed to darker staining and increased calcified nodule formation (Figure 5C). In addition, the ALP staining and activity test showed light staining and reduced ALP activity in the miR-34c inhibitor + SP600125 treatment group compared with miR-34c inhibitor + DMSO treatment (*p* < 0.05). This was also in line with the results observed following the oe-STC1 + SP600125 treatment when compared with oe-STC1 + DMSO treatment (*p* < 0.05). Conversely, upregulation of STC1 resulted in promoted ALP staining and activity (Figure 5D). Taken together, miR-34c could inhibit the osteogenic differentiation and calcification of VICs by suppressing STC1 to block the JNK signal pathway, so as to affect CAVD.

## Discussion

Calcific aortic valve disease is a process that involves varies kinds of pathologic changes. VICs are the predominant cell type in the heart valve and are involved in maintaining normal valve structure and function (Zhang et al., 2014). The miR-34 family, which includes miR-34a/b/c, is a group of well-known, non-coding RNAs, which could regulate gene expression after transcription (Imani et al., 2018). STC1 mRNA expression is high in perichondrial cells, periosteal cells and osteoblasts during the formation of endochondral bone (Yoshiko et al., 2002). Our study identifies a new direction for the treatment of CAVD, in which miR-34c suppresses STC1 and the JNK signaling pathway, leading to the alleviation of CAVD.

We first determined that miR-34c was downregulated in CAVD, and that up-regulation of miR-34c could alleviate the symptoms associated with CAVD. miRNAs were shown to regulate the shift of phenotype through distinctive miRNA programs with signatures that were cell-specific, which could initiate smooth muscle cells calcification (Leopold, 2014). Low expression of miR-34b/c was found in vascular smooth muscle cell (VSMC) calcification, and overexpression of miR-34b/c alleviated VSMC calcification (Hao et al., 2016). In addition, we found that elevated STC1 expression exaggerated CAVD and up-regulation of miR-34c inhibited CAVD, suggesting that miR-34c could target and inhibit the expression of STC1. One study showed the mRNA expression of STC1 was relatively high in colonies of maturing osteoblast co-expressed with alkaline phosphatase, bone sialoprotein and osteocalcin (Yoshiko et al., 2003). Another study demonstrated that miR-101b targeted STC1 (De Martino et al., 2009). This may further support the negative correlation between STC1 and miR-34c and their regulation on the CAVD.

We also found that upregulation of miR-34c could inhibit osteogenic differentiation and calcification in VICs, and might alleviate the symptoms of CAVD, as evidenced by repressed expression of BMP2 and osteocalcin as well as decreased formation of calcified nodules. Our findings are supported by the fact that CAVD is an active regulatory process connected with osteoblast-like phenotype (Rajamannan et al., 2003), and that the miR-34 family can regulate the proliferation and/or differentiation of osteoblasts (Wei et al., 2012). Overexpression of STC2 inhibited phosphate-induced calcification in aortic vascular smooth muscle cells (Takei et al., 2012). miR-204 could negatively regulate osteogenic differentiation by inhibiting Runx2, thus suppressing osteoblast-related genes expression such as BMP2-induced alkaline phosphatase and osteocalcin (Wang et al., 2015). In addition, the expression of miR-141 was associated with BMP2 signaling inhibition and calcification *in vitro* (Yanagawa et al., 2012). Combined with the findings above, STC1 was identified as a downstream target of miR-34c, and miR-34c could inhibit VIC osteogenic differentiation and calcification through binding to STC1.

Finally, our study also found that miR-34c could affect CAVD by targeting the STC1-mediated JNK signaling pathway. Normally, osteoblast differentiation is inhibited by the impaired JNK pathway, and JNK could be activated after cells are exposed to chemotherapeutics (Lagadinou et al., 2008). We found that activation of the JNK pathway was inhibited by miR-34c through its targeting of STC1. A previous study indicated that JNK signal pathway could be inhibited by recombinant STC1 protein (Chan et al., 2017). The activation of p53-mediated JNK1 was essential in the miR-34a induction by deoxycholic acid (Ferreira et al., 2014). Another study demonstrated that the inflammatory response could be inhibited by miR-92a through targeting mitogen-activated protein kinase kinase 4/JNK/c-Jun pathway (Lai et al., 2013). Furthermore, another research demonstrated that miR-206 played an important role in regulating normal convergent and extension movements through its regulation of the JNK pathway (Liu et al., 2012).

## Conclusion

In conclusion, our research indicates that miR-34c could inhibit osteogenic differentiation and calcification of VICs by targeting STC1 to suppress JNK signaling pathway (Figure 6), hence providing a potential therapeutic target for the CAVD.

**FIGURE 6:** MiR-34c binds to STC1 to inhibit the activation of the JNK pathway, resulting in the suppression of the osteogenic differentiation and calcification degree in VICs.

## Data Availability Statement

The raw data supporting the conclusions of this article will be made available by the authors, without undue reservation.

## Ethics Statement

Technical problem while retrieving the ethics statement verify manually.

## Author Contributions

LY, XZ, and YN designed the study. DW, YT, and ZC collated the data, carried out the data analyses, and produced the initial draft of the manuscript. ML, HZ, and DL contributed to drafting the manuscript. All authors read and approved the final manuscript.

## Conflict of Interest

The authors declare that the research was conducted in the absence of any commercial or financial relationships that could be construed as a potential conflict of interest.

## Footnotes

1 https://www.ncbi.nlm.nih.gov/geo/
